# Valproic Acid Inhibits Peripheral T Cell Lymphoma Cells Behaviors via Restraining PI3K/AKT Pathway

This article has been retracted.

**DOI:** 10.1155/2022/7350489

**Published:** 2022-08-05

**Authors:** Zhiqiang Peng, Jianping Xiong, Hanzhi Dong

**Affiliations:** ^1^Department of Oncology, The First Affiliated Hospital of Nanchang University, Nanchang 330006, Jiangxi, China; ^2^Department of Lymphatic Hematology and Oncology, Jiangxi Cancer Hospital, Nanchang 330029, Jiangxi, China; ^3^General Department of Oncology, Jiangxi Cancer Hospital, Nanchang 330029, Jiangxi, China

## Abstract

**Objective:**

Alproic acid (VPA) is a clinic antiepileptic drug. Antitumor role of VPA has been studied. The aim of this study was to clarify the treatment effect and potential mechanism of VPA on peripheral T cell lymphomas (PTCLs).

**Materials and Methods:**

Hut 78 cells were obtained from the Shanghai Cell Bank, Chinese Academy of Sciences, and randomly divided into six groups: control, VPA (8 mM), empty vector (NC), miR-3196 mimics, miR-3196 inhibitor, and VPA + miR-3196 mimics groups. CCK-8 assay was performed to clarify the regulative role of VPA on cell proliferation. Flow cytometry was applied to determine the apoptotic rate and ROS levels. miR-3196 was tested by RT-qPCR. Western blot was used to test the level of p-PI3K and p-AKT. Biochemical experiments were used to detect changes in the content of ATP, lactate level, and glucose content. Electron microscopy was used to show the structure of mitochondria in Hut 78 cells.

**Results:**

VPA greatly promoted the expression of miR-3196 and inhibited cell proliferation in a dose-dependent manner. Compared with the NC group, the cell apoptosis rate, Bax and cleaved-caspase-3 expression, lactate level, ROS expression, and glucose content in the VPA group were significantly increased (*P* < 0.05), and cell proliferation, ATP production, and the expression of Bcl-2, p-PI3K and p-AKT was decreased significantly (*P* < 0.05). The role of mir-3196 mimics is similar to VPA. While, the miR-3196 inhibitor had the opposite effect to VPA and mimics. The combination of VPA and miR-3196 mimics has the most obvious effect.

**Conclusion:**

VPA can inhibit the proliferation of Hut 78 cells and promote cell apoptosis and the structure and dysfunction of mitochondria by regulating the activity of the PI3K/AKT pathway.

## 1. Introduction

Peripheral T cell lymphomas (PTCLs) are a group of heterogeneous lymphoproliferative diseases caused by mature T cells or natural killer cells, accounting for about 10%–15% of the total malignant lymphoma [1–3]. The incidence of PTCL has distinct geographical and ethnic characteristics, accounting for 25%–30% of non-Hodgkin lymphoma (NHL) incidence in the oriental population [4–6], which is significantly higher than 10%–15% reported in European and American countries [7, 8]. As PTCL has diverse clinical symptoms, PTCL could affect upper digestive tract to induce esophageal stricture and dysphagia [9]. Tongue could also be the target tissue of lymphoma [10]. The symptoms of digestive lymphoma are similar to that of Crohn's disease [11]. It is prone to missed diagnosis and misdiagnosis. The main frontline therapies include brentuximab vedotin [12], histone deacetylase inhibitors [13], pralatrexate [14], mogamulizumab [15], alemtuzumab [16], lenalidomide [17], azacitidine [18], PI3Ki [19], and consolidative stem cell transplantation [20]. However, its overall treatment efficacy is still poor, with a 5-year survival of only 10%–30% [21]. Further studies are needed to investigate the pathogenesis of PTCLs, which are of great significance for the prevention and treatment of PTCLs.

Alproic acid (VPA) is a commonly used antiepileptic drug in clinics. Due to its histone deacetyltransferase inhibitor function, its potential antitumor effect has been widely valued. Many studies have shown that VPA has a certain antitumor effect [22–24]. In the combined treatment research of VPA and other chemotherapeutics, it is found that VPA itself has the effect of inhibiting tumor cells, and it can also increase the sensitivity of tumor cells to certain chemotherapeutic drugs and reduce the drug resistance of tumor cells [25, 26]. VPA can also regulate the expression of miRNAs in tumor cells to play an antitumor role [27]. However, the effects of VPA on miRNAs in peripheral T lymphocytic lymphoma and their specific regulatory mechanisms are currently poorly studied and still need further study.

miRNAs have been widely studied in various disease. They are a group of short noncoding RNA that inhibits the function of target gene via binding to its mRNA [28]. The role of miRNAs in PTCLs has been confirmed by some studies. miRNA-126-3p and miR-145-5p are increased in PTCL and perform T cell migrative regulation [29]. Hsa-miR-372-5p regulates NLRP3 inflammasome activation via targeting in NK/T cell lymphoma [30]. miR-548 could inhibit the progression of NK/T cell lymphoma via targeting FOXO1 [31]. These evidences reveal the potential regulation role of miRNAs in PTCL. However, the role of miRNAs in PTCL is still not fully clarified. The involved miRNAs and their target genes need to be uncovered. miR-3196 has been confirmed to regulate lung adenocarcinoma cell migration and invasion via Sox12 [32]. miR-3196 could regulate cell proliferation, migration, and EMT (epithelial-mesenchymal transition) via STRN4 in drug-resistant cells of liver cancer [33]. However, the role of miR-3196 in PTCL has not been explored. Whether miR-3196 was the downstream gene in VPA treating needs to be verified.

In this study, we used VPA to process Hut 78 cells and then observed the effects of VPA on the proliferation, apoptosis, mitochondrial structure, and function of Hut 78 cells and further explore whether its effect is achieved by regulating the PI3K/AKT pathway.

## 2. Materials and Methods

### 2.1. Cell Culture

To detect the role of VPA PTCL cells, Hut 78 cells (TCHu206, Shanghai Cell Bank, Chinese Academy of Sciences), a commonly used T cell lymphoma cell in tumor research studies [34], were cultured and in vitro analysis was conducted. These cells were purchased from IMDM (SH30228.01B; Hyclone), adding 20% fetal bovine serum (FBS, 10270-106; Gibco) was applied to culture the cell in vitro. The cells were cultured in a 37°C constant temperature incubator (5% CO_2_). The culture medium was changed every day.

### 2.2. Cell Transfection

The sequence of miR-3196 (GI: 301171776) was checked at the NCBI database. miR-3196 mimics (5′-CGGGGCGGCAGGGCCUC-3′) or inhibitor (5′-CGGGGCGGCAGGGCCUC-3′) was transported into the cell with Lipofectamine 2000. The transfection was conducted according to the manufacturer's instructions. 24 hours before transfection, inoculate 1 × 10^5^ cells in 500 *μ*L medium and adjust the cell number to 6 × 10^5^/well during transfection. siRNA (1 *μ*l, 10 *μ*M) was diluted with Opti-MEM (50 *μ*L). Then, 5 *μ*l Lipofectamine® RNAiMAX was added into 50 *μ*L Opti-MEM. These reagents were mixed and maintained in the fridge (4°C, 5 minutes). Finally, the cells were kept in an incubator at 37°C and 5% CO_2_ for 24 hours.

Cells were intervened with miR-3196 mimics or miR-3196 inhibitor for 48 h and, respectively, divided into six groups: control, VPA, empty vector (NC), miR-3196 mimics, miR-3196 inhibitor, and VPA + miR-3196 mimics groups.

### 2.3. Cell Counting Kit-8 (CCK-8)

To detect the cell viability, CCK-8 assay was used. The suspending cells were cultured in 96-well plates at a density of 1 × 10^4^ cells/ml with IMDM adding 20% FBS for 48 h. Then, 10 *μ*l CCK-8 reagent was added to each well of the plates. The cells with CCK-8 were incubated at 37°C for 4 h. The optical density (450 nm) was determined with a microplate reader (Multiskan FC, Thermo, USA).

### 2.4. Flow Cytometry

After culturing for 48 h, the cell samples from different groups were harvested, added in 1 ml precooled PBS, and centrifuged at 1000*g* for 5 min. The supernatant was discarded. The cells were resuspended with cold PBS, and Annexin V-FITC and PI were added. The cell apoptotic rate and ROS level of cells were analyzed using flow cytometry according to the manufacturer's instructions, and the data were analyzed by flow cytometry (Beckman Coulter, USA).

### 2.5. The Detection of Glucose, A095-1, and A019-2

To detect the level of lactic acid (A019-2), ATP (A095-1), and glucose (F006), the assay kits were brought from Nanjing Jiancheng Bioengineering Institute. The experiments were conducted according to the manufacturer's instruction.

### 2.6. Transmission Electron Microscopy (TEM)

After rinsing the cells with cold PBS for three times, 2.5% glutaraldehyde was applied to prefix the cells (4°C, 30 min). Then, 1% osmic acid was used to fix the cells for 1 h. Then, after dehydrating, the samples were incubated in acetone and epoxy mixture (1 : 1) at 40°C for 6 h. After further fixing with pure epoxy resin (40°C, 4 h), the samples were embedded and sliced. The slices were double stained and stained with lead citrate for 15 min. The slices were rinsed with double-distilled water. Finally, the mitochondria ultrastructure was recorded with TEM (HT7700, Hitachi).

### 2.7. Western Blot Analysis

The total proteins from cells were extracted, and the concentration was measured by the BCA protein assay kit (Beyotime, China). Total protein was separated in SDS-PAGE (12%). The proteins were then transferred to the PVDF membrane. The membranes were blocked with a blocking buffer (5% nonfat milk, 0.05% Tween-20) which was used to block the membranes. Then, the membranes were labeled with primary antibody including anti-Bad antibody (1 : 1000, MAB37156, Bioswamp), anti-Bcl-2 antibody (1 : 1000, PAB33482, Bioswamp), anti-cleaved-caspase-3 antibody (1 : 1000, MAB37300, Bioswamp), anti-PI3K antibody (1 : 1000, PAB30009, Bioswamp), anti-AKT antibody (1 : 1000, PAB34089, Bioswamp), and anti-GAPDH antibody (1 : 1000, PAB36264, Bioswamp). The membranes were rinsed with PBS/Tween-20 three times. Then, the membranes were further labeled with horseradish peroxidase-conjugated secondary goat anti-rabbit IgG (1 : 10000, SAB43711, Bioswamp) for 2 h at room temperature. The blots were visualized by enhanced chemiluminescence color detection (Tanon-5200, TANON, China).

### 2.8. Quantitative Real-Time Polymerase Chain Reaction (qRT-PCR)

The total RNAs of the cultured cell were extracted with TRIzol (Beyotime, China) kit. The cDNAs were synthesized with the reverse transcriptase kit (TAKARA, USA). RT-qPCR was conducted with the SYBR Green PCR Kit (KM4101, KAPA Biosystems) on the real-time system (Bio-Rad. The 2^−△△Ct^ method was used to analyze the expression of the RNAs. The primers sequences are given in Table 1 (Nanjing Kingsy Biotechnology Co., Ltd.) (Table 1).

### 2.9. Statistical Analysis

The data were recorded as the mean ± standard deviation. *t* tests were used to analyze the differences between two groups. One-way ANOVA was used to analyze differences between groups. SPSS 22 statistical software was used to conduct statistical analysis. *P* < 0.05 was considered statistically significant.

## 3. Results

### 3.1. VPA Promotes miR-3196 Expression and VPA and miR-3196 Promote Cell Proliferation in a Synergistic way

We first detected miR-3196 expression in Hut 78 cells after different concentrations of VPA intervention. Compared with the control group, different doses of VPA could significantly increase the expression of miR-3196 (*P* < 0.05) (Figure 1(a)). CCK-8 analysis was conducted to clarify the effect of VPA on the Hut 78 cell proliferation. The results showed that compared with the control group, the cell proliferation rate in the VPA group (0 mM, 0.5 mM, 1 mM, 2 mM, 4 mM, 8 mM, 16 mM, and 32 mM) [35] was significantly reduced (*P* < 0.05), and the 32 mM VPA group had the lowest cell proliferation rate (Figure 1(b)). The CCK-8 experiment showed that IC50 of VPA on Hut 78 cells was 16 mM. Therefore, we use 0.5 IC50 (8 mM) as the VPA intervention concentration for subsequent experiments. The transfection efficiency of miR-3196 mimics/inhibitor was further detected by RT-qPCR (Figure 1(c)). The expression of miR-3196 in the miR-3196 mimics group was evidently increased compared with the control group (*P* < 0.05). The expression level of miR-3196 was significantly decreased in the miR-3196 inhibitor group compared with the control group (*P* < 0.05). These data suggested that miR-3196 mimics and miR-3196 inhibitor were successfully transfected. As shown in Figure 1(d), the cell proliferation rate of the VPA group was greatly reduced compared with that in the control group (*P* < 0.05). Compared with the NC group, the cell proliferation rate was decreased in the miR-3196 mimics group and VPA + miR-3196 mimics group (*P* < 0.05). While, it was increased in the miR-3196 inhibitor group (*P* < 0.05).

### 3.2. VPA and miR-3196 Promote Cell Apoptosis in a Synergistic way

Flow cytometry was performed to determine the apoptotic rate of cultured Hut 78 cells. As shown in Figure 2(a), the apoptotic rate of the VPA, miR-3196 mimics, and VPA + miR-3196 mimics group was greatly promoted compared with that in the control group (*P* < 0.05). The apoptotic rate of the miR-3196 inhibitor group was evidently inhibited compared with that in the control group (*P* < 0.05). The apoptotic rates of the miR-3196 mimics group and VPA + miR-3196 mimics group were greatly promoted compared with that in the NC group (*P* < 0.05), while the apoptotic rate of the miR-3196 inhibitor group was evidently reduced (*P* < 0.05). We further detected the expression of related apoptotic proteins, and the results showed that compared with the control, Bax and cleaved-caspase-3 expressions were significantly increased in the VPA, miR-3196 mimics, and VPA + miR-3196 mimics group (*P* < 0.05), and the level of Bcl-2 was greatly reduced in the VPA, miR-3196 mimics, and VPA + miR-3196 mimics group (*P* < 0.05) (Figure 2(b)). Compared to the NC group, the expression of Bax and cleaved-caspase-3 in the miR-3196 mimics group and VPA + miR-3196 mimics group increased significantly (*P* < 0.05), while Bcl-2 expression in these groups was evidently inhibited (*P* < 0.05).

### 3.3. VPA and miR-3196 Affect Mitochondrial Morphology, ROS Production, and Cell Metabolism

In Figure 3(a), TEM was conducted to show the impact of VPA and miR-3196 on mitochondrial structure of Hut 78 cells. The shape of mitochondria in the control group was oval or rod with neat mitochondria cristae. The cristae lumen was not dilated. In the VPA group and miR-3196 mimics group, the swelling and deformation of mitochondria showed spherical structure, the internal cristae decreased, and some vacuolization. Compared with the control group, the production of ROS was greatly promoted in the VPA group (*P* < 0.05). Compared with the NC group, ROS levels in miR-3196 mimics and VPA + miR-3196 mimics groups were significantly increased (*P* < 0.05), while ROS level was significantly decreased (*P* < 0.05) in the miR-3196 inhibitor group (*P* < 0.05) (Figure 3(b)). We further tested the effects of VPA on the cell metabolism. As the result shown in Figure 3(c), compared with the control group, the ATP production in the VPA group decreased (*P* < 0.05), and the lactate level and glucose content increased (*P* < 0.05). Compared with the NC group, the ATP production in the miR-3196 mimics group and VPA + miR-3196 mimics increased (*P* < 0.5) and the lactic acid content and glucose content decreased (*P* < 0.5).

### 3.4. VPA and miR-3196 Regulate PI3K/AKT Pathway

To study whether VPA and miR-1396 play its role through the PI3K/AKT pathway, we used Western blot to detect key proteins in the PI3K/AKT pathway. The level of p-PI3K and p-AKT were decreased in the VPA group compared with that in the control group (*P* < 0.05). Compared with the NC group, the expression of p-PI3K and p-AKT was decreased in the miR-3196 mimics group and VPA + miR-3196 mimics group (*P* < 0.05) and increased significantly in the miR-3196 inhibitor group (*P* < 0.05). These results suggested VPA and miR-3196 can play a protective role by inhibiting the PI3K/AKT pathway (Figure 4).

## 4. Discussion

Peripheral T cell lymphoma (PTCL) is a type of heterogeneous lymphoproliferative diseases that affect multiorgan including the digestive system. When PTCLs occur in the digestive system, dysphagia, digestive tract stenosis, and other type of symptoms like Crohn's disease could occur [9–11]. Clarifying the pathogenic mechanism of PTCLs is important to the development of effective therapeutic methods.

Aberrant epigenetic dysregulation, including DNA methylation, histone modification, chromatin remodeling, gene imprinting, and random chromosome (x) inactivation, plays a key role in tumorigenesis. Histone deacetylases (HDACs) and histone acetyltransferases (HATS) are involved in epigenetic regulation of genes by controlling the acetylation status of lysine residues in the histone tail [36]. HATS acetylate histone tails to form an “open” chromatin structure that facilitates the execution of gene transcription. In contrast, HDACs control the deacetylation of histone tails, which holds chromatin in a “closed” state and causes the expression silencing of relevant genes [37]. Normally, HDACs and hats are in a dynamic equilibrium between each other, and the disruption of their balance is closely related to tumor initiation and progression. HDACs, which regulate the deacetylation of histones and certain nonhistone proteins, including the activation of tumor initiation related transcription factors as well as posttranslational modifications of key proteins including tumor suppressor genes [38–40], have emerged as a potential anticancer target because of their close association with cancer cell proliferation, apoptosis, differentiation, migration, and metastasis [40]. Studies have found that VPA is able to exert its anticancer effects by altering the histone acetylation levels of tumor cells, while also downregulating the expression levels of the antiapoptotic protein survivin, counteracting its antiapoptotic effect, and playing a role in inducing tumor cell apoptosis. Thus, in this experiment, we first detected the effect of VPA on the proliferation and apoptosis of PTCLs. The results showed that compared with the control group, the treatment of VPA can significantly inhibit the proliferation of Hut 78 cells and promote its apoptosis, suggesting that VPA can significantly inhibit the proliferation of PTCLs and promote cell apoptosis.

Mitochondria are an important source of energy in cells, and their morphology is a dynamic change process in the cell process. Mitochondria are extremely vulnerable to the attack of reactive oxygen species, which leads to the breakdown of the dynamic balance of mitochondrial fission and polymerization, and ultimately leads to cell apoptosis [41–44]. Studies have found [45] that histone deacetylase inhibitors can inhibit the formation of reactive oxygen species in tumor cells, promote the activation of caspase-8, caspase-9, caspase-3 and PARP, and ultimately lead to cell apoptosis. However, it is rarely reported whether VPA regulates the mitochondrial function of T lymphocyte tumors and promotes cell apoptosis. Thus, in this experiment, we first detected the expression of ROS in each group; the results showed that the expression of ROS in the VPA group was significantly increased compared to the control, suggesting that VPA can effectively promote the expression of ROS. We further observed the effect of VPA on mitochondrial structure of Hut 78 cells and found that the mitochondria in the control group were oval or rod-shaped, and the cristae in the mitochondria was neat, and the lumen of the cristae was not dilated. In the VPA group and miR-3196 mimics group, the swelling and deformation of mitochondria showed spherical structure, the internal cristae decrease, and some vacuolization.

The PI3K/AKT/mTOR signaling pathway is a classical pathway that regulates cell growth and proliferation and is closely related to a variety of diseases. In the previous experiments of this study, we found that VPA could inhibit the proliferation of Hut 78 cells, promote cell apoptosis, and the structure and dysfunction of mitochondria. Therefore, we speculate that VPA may be achieved by regulating the PI3K/AKT pathway. The results showed that the expression of p-PI3K and p-AKT decreased in the VPA group compared to the control, prompting that VPA can inhibit the activity of the PI3K/AKT pathway. There are some limitations of this study. The target gene of miR-3196 could be confirmed. The animal verification is also suggested. We will complete these in further study.

In conclusion, VPA can inhibit the proliferation of Hut 78 cells and promote cell apoptosis and the structure and dysfunction of mitochondria, and its effect may be achieved by regulating the activity of the PI3K/AKT pathway. VPA could be a potential treatment drug on PTCLs.

## Figures and Tables

**Figure 1:** VPA promotes miR-3196 expression, and VPA and miR-3196 promote cell proliferation in a synergistic way. (a) RT-qPCR used to detect miR-3196 expression. ((b) and (d)) CCK-8 used to detect Hut 78 cell proliferation after 48 hours of valproic acid intervention. (c) miR-3196 expression detected by RT-qPCR. ^*∗*^*P* < 0.05 vs. control; ^#^*P* < 0.05 vs. NC. *N*  = 3.

**Figure 2:** VPA and miR-3196 promote cell apoptosis in a synergistic way. (a) Cell apoptosis detected by flow cytometry. (b) Expression of Bcl-2, Bax, and cleaved-caspase-3 tested by Western blot. ^*∗*^*P* < 0.05 vs. control; ^#^*P* < 0.05 vs. NC. *N*  = 3.

**Figure 3:** VPA and miR-3196 affect mitochondrial morphology, ROS production, and cell metabolism. (a) Mitochondrial morphology examined by electron microscopy (scale bar = 1 mM). (b) ROS level detected by flow cytometry. (c) ATP production, lactate level, and glucose content observed by biochemical analysis. ^*∗*^*P* < 0.05 vs. control; ^#^*P* < 0.05 vs. NC. *N*  = 3.

**Figure 4:** VPA and miR-3196 regulate the PI3K/AKT pathway. Expression of p-PI3K and p-AKT protein observed by Western blot. ^*∗*^*P* < 0.05 vs. control; ^#^*P* < 0.05 vs. NC. *N*  = 3.

**Table 1:** Primer sequences.

Primers	Sequence (5′-3′)
miR-3196-F	GGGCGGGGCGGCAGGG
miR-3196-R	AACTGGTGTCGTGGAGTCGGC
U6-F	CTCGCTTCGGCAGCACA
U6-R	AACGCTTCACGAATTTGCGT

## Data Availability

The data used to support this study are available from the corresponding author upon request.
